# Diagnosis and Treatment Rules of Chronic Kidney Disease and Nursing Intervention Models of Related Mental Diseases Using Electronic Medical Records and Data Mining

This article has been retracted.

**DOI:** 10.1155/2021/5187837

**Published:** 2021-12-10

**Authors:** Yanli Wang, Yueyao Sun, Na Lu, Xuan Feng, Minglong Gao, Lihong Zhang, Yaping Dou, Fulei Meng, Kaidi Zhang

**Affiliations:** ^1^Department of Mental Health, The First Hospital of Hebei Medical University, Shijiazhuang, China; ^2^Department of Hepatobiliary Surgery, The First Hospital of Hebei Medical University, Shijiazhuang, China; ^3^Department of Emergency, The First Hospital of Hebei Medical University, Shijiazhuang, China; ^4^Department of Nephrology, The First Hospital of Hebei Medical University, Shijiazhuang, China; ^5^Department of Respiratory Medicine, First Hospital of Hebei Medical University, Shijiazhuang, China

## Abstract

**Objective:**

On the basis of electronic medical records, the data mining technology was adopted to explore the law of chronic kidney disease (CKD) and the intervention mode of mental health of patients.

**Methods:**

Based on the electronic medical records, the corresponding data extraction, database establishment, and data cleaning of CKD were performed. After that, the related data analysis, frequency analysis, cluster analysis, and nonparametric analysis were used to explore the laws of CKD diagnosis and treatment and nursing intervention mode of mental illness. The most common causes of CKD were chronic glomerulonephritis (43.76%), aristolochic acid nephritis (16.34%), diabetic nephritis (12.87%), and hypertensive nephritis (11.58%). The major treatment method for end-stage patients was alternative therapies, accounting for 46%. Compared with the depression score before intervention, that of the patients after the mindfulness therapy (50.99 ± 9.77 vs. 47.01 ± 9.33, *P*=0.024 < 0.5) and target behaviour nursing intervention (52.21 ± 8.12 vs. 48.01 ± 9.33, *P*=0.032 < 0.05) was obviously decreased.

**Conclusion:**

The data mining technology based on electronic records showed a good application prospect in the analysis of the diagnosis and treatment of CKD; and target behaviour nursing and mindfulness intervention were effective psychological intervention models.

## 1. Introduction

Chronic kidney disease (CKD) is a type of clinical syndrome with primary or secondary renal injury as the main clinical feature. Its further development will further cause irreversible damage to the kidney tissue and function, which will further cause the retention of metabolites and poisons, the imbalance of water and electrolyte, acid-base, endocrine disorders, and other characteristics, and lead to chronic renal failure [1]. The causes of CKD treatment are complex and diverse. The most common type of CKD in China is IgA-based primary glomerulitis, followed by hypertension renal arterioles, diabetic nephropathy, lupus nephritis, chronic pyelonephritis, and polycystic kidney disease. At present, the treatment of CKD is mainly based on the treatment of research and development diseases to eliminate the reversible factors of renal function deterioration [2]. The most common treatment method is the use of drugs such as hormones, cytotoxic drugs, cyclosporine A, and diuretics. However, the long-term use of these drugs often produces adverse reactions and complications, and some patients may suffer from drug insensitivity or dependence. These factors make many patients experience recurrent disease, which is very unfavourable for the treatment and prognosis of the disease [3–5]. In addition, some auxiliary treatment methods are generally added according to the actual situation of the patient in clinical practice, such as nutritional therapy, antihypertensive therapy, control of urine protein, treatment of renal anemia, renal osteopathic medicine, correction of water electrolyte and acid-base balance disorders, prevention and treatment of cardiovascular disease, control of infection, promotion of intestinal excretion of uremic poisons, and kidney replacement [6, 7]. All in all, there are currently no specific effective treatment methods and drugs for the treatment of CKD.

With continuous development and progress of network technology and information technology, the degree of informatization of hospitals has gradually been comprehensive and in-depth. The electronic medical records system belongs to the most important part of the system [8]. According to the Electronic Medical Records Basic Framework and Data Standards promulgated by the former Ministry of Health in December 2009, electronic medical records are defined as the data integration system created, stored, and used by medical institutions in form of electronic medical records. It can comprehensively record the complete and specific clinical information generated by the patient during the medical treatment process [9]. Such information is of great significance for clinical research. With the widespread use of electronic medical records, the amount of data in the electronic medical records database has grown rapidly. But the ability to deeply mine these data, extract effective information, and extract effective patterns is insufficient in current days [10]. Traditional database retrieval and statistical methods can no longer meet our current data extraction and analysis needs. In this context, the application of data mining in hospital information systems has become a research hotspot in recent years. Among many data mining methods, association rule data mining has been widely recognized and concerned, and it is mainly divided into Apriori algorithm and FP-Growth algorithm. In recent years, the above two algorithms have been widely used in all walks of life and have been applied to the analysis of electronic medical records [11]. Relevant studies have shown that the use of association rule data mining and analysis of electronic medical records can not only analyse the pathogenic factors of diseases, the law and trend of disease development, and the relationship between different medication behaviours and treatment results, but also provide references and basis for treatment and diagnosis by the doctors and provide references for operating rules of the hospital obtained from data analysis [12].

A large amount of clinical data show that CKD has a longer course, poor prognosis, and higher treatment costs [13]. In this context, the risk of patients suffering from mental illnesses is greatly increased. Depression is one of the most common psychological and physical reactions in patients with chronic nephritis. Patients often show indifferent attitudes towards surrounding things, loss of appetite, very low mood, less speech, and sleep disturbances. Some patients do not follow the doctor's advice during treatment, refuse treatment, or even commit suicide. In addition, mental illnesses such as depression can also cause a series of endocrine dysfunction and reduce the immune capacity of body. These are extremely detrimental to the prognosis and outcome of the disease. At present, there are a few studies on mental illnesses related to chronic disease patients and effective nursing interventions in China. A statistics and analysis are of great significance to the formulation of nursing intervention programs for related diseases.

In this study, the rules of diagnosis and treatment of CKD patients and the nursing model of related mental illnesses were explored based on electronic medical records and data mining technology. It was expected to provide reference and basis for the diagnosis and treatment of clinically related diseases.

## 2. Materials and Methods

### 2.1. Research Object

168 electronic medical records of patients with CKD from the Department of Nephrology of the First Hospital of Hebei Medical University in the past three years were the research objects. The selected electronic medical records had to meet the following requirements: the records included complete information, including age, gender, date of visit, and relevant examination results; they were electronic records of patients with CKD; and the patients included in the medical record had not died and can communicate normally. The exclusion criteria were defined as follows: the medical records with missing information and incomplete data, such as medication information and electronic medical records of missing important examination results; and the kidney disease recorded in the electronic medical record did not belong to the medical history of CKD, such as the medical history of patients with renal failure caused by other diseases.

### 2.2. Data Extraction

The data of electronic medical records is huge, so the data has to be extracted. It categorized and extracted some of the attribute values that were valuable for the relevant research of this study according to the order of electronic medical records. The specific main database attribute values were as follows: medical history, examinations and inspections, and surgery and diagnosis. The attribute in the medical history was an explanation of the patient's condition before and at the time when he came to the hospital. This part of the annual content was mainly extracted from the main statement, current medical history, past history, personal history, and family history in electronic medical records, including symptoms at the time of admission, prehospital conditions, health conditions, living habits, mental conditions, and genetic history. The attributes in the examinations and inspection were mainly to explain the relevant inspections during the treatment of the patient. This part of the attribute was mainly extracted from the physical examination and inspection and disease course records in electronic medical records, such as blood pressure, pulse, respiration, blood routine (multiple times), liver and kidney function, and other attributes. Most of these attributes had multiple subattributes and multiple check values, so multiple tables needed to be established to associate with them. The surgery and diagnosis include patient dialysis, kidney B-ultrasound, and kidney transplantation.

### 2.3. Establishment of Dataset

The extracted data cannot be directly stored in the database, so it is necessary to define the data type of each part of the extracted information, convert it into a data form that can be processed by the computer, and then store it in the database. For the digital information in the text, such as body temperature, respiration, blood pressure, and pulse, it can be converted into digital fields and stored directly in the database. But most medical information has multiple choices. Therefore, it is necessary to define an index item when this part of information is dealt with. In the table dedicated to this type of information, each possible value is represented by the index item. The following items were the relationship between the partial indicator and the corresponding value. The symptoms included back pain, thirst, and weakness or not (1 for no and 2 for yes). The personal history included smoking and alcohol drinking or not (1 for no, 2 for yes, and 3 for stopped). The family history included genetic history of kidney disease and hyperemia or not (1 for no and 2 for yes). For laboratory test values, 1 meant the value was within the required range, and 2 and 3 meant the value was higher and lower than the required range, respectively. The data was processed and stored in the database.

### 2.4. Data Clearing

The original data extracted and stored in the database is incomplete and inconsistent, which can be solved by filling in vacant values, correcting illegal values, and correcting data inconsistencies. For attribute items with no data value, it can define a vacant value according to the meaning of the data item for most data and then use it to replace the vacant value. If the blood routine prompts “N73.4%, L18.2%, HCT36.0%, and MPV13.8%,” it should fill in the corresponding data drawn in the blood routine table, and the value of the experimental check value range is filled in 2 (high), 3 (low), 3, 2, 1, respectively. The data in the electronic case have a certain limited range, and the data outside the limited range are all illegal data. If these data are directly used for processing, they will cause large deviations in the processing results and reduce processing efficiency. Generally, the reason for the occurrence of illegal data is the writing error by doctor. For example, the number “1” and the letter “l,” the number “0” and the letter “O” are often confused, and it is generally difficult to detect and find manually, so some special methods have to be adopted to recover the correctness. For example, when “PAl36 mg/L” is extracted, it has to separate the characters, numeric characters, and units firstly and assign values to variables s1, s2, and s3, respectively, so that s1 = PAl, s2 = 36, and s3 = mg/L. Then, it can search for a record matching s1 in the blood lipid and electrolyte category of the dictionary database, determine that the last character of s1 is “l,” and convert “l” into a number character “1.” After it is added to the variable s2 and the character is converted to a number, “136” is obtained. The original data not only shows incompleteness, but also shows inconsistency in some data. There is a correlation between some data, and this correlation can be used to solve the data inconsistency. In this study, the data protocol technology was adopted to deal with inconsistent data. Protocol technology mainly involves symptoms, medical history, personal history, and auxiliary examination results. Some attributes were undertaken as examples to illustrate the specification method as follows. The attributes of the symptom part include back pain or not (symptom_1), thirst or not (symptom_2), weakness or not (symptom_3), poor sleep or not (symptom_4), nocturia or not (symptom_5), edema or not (symptom_6), and other (symptom_7). For the typical symptoms of CKD (waist and knee soreness), the above attributes can be reduced to a typical symptom attribute (symptom_0) with disease, disease history (disease-his), and symptom history (symptom_his). Its attribute values 1, 2, and 3 represent typical, atypical, and others, respectively. The new attribute value after the protocol is not completely equal to the value of the attribute symptom_2 or symptom_3, so the value of other attributes can be used to correct the inconsistency of these data. The correction method was as follows:

  if (disease_*∗* = “CKD” and disease_his_*∗* > 0)
  then symptom_0 = 1//typical
  else if symptom_*∗* = 2 then symptom_0 = 1//typical
  else if (symptom_2 = 2 or symptom_3 = 2) then symptom_0 = 1//typical
  else if (symptom_5 = 2 and symptom_his >0) then symptom_0 = 1//typical
  else if (symptom_7 = 2 and symptom_his_7 > 0) then symptom_0 = 2//not typical
  else symptom_0 = 2//other

Asterisk represents all suffix numbers of this type of attribute.

The attributes of the disease included known and diagnosed disease_1, disease_2, disease_3, disease_4, and disease_5. In this study, the main diagnoses related to coronary heart disease (CHD) were taken. The disease history attribute is reduced to the typical disease history attribute disease_0, and the attribute values 1, 2, and 3 indicated that they were “confirmed,” “correlated,” and “uncorrelated,” respectively. The logical relationship of the attribute disease_0 was as follows:

  if (disease_*∗* = “CKD”or disease_*∗* = “renal failure”)
  then disease_0 = 1//confirmed
  else if (disease_*∗* = “hypertension” or disease_*∗* = “diabetes” or disease_*∗* = “hyperlipidemia”)
  then disease_0 = 3//correlated
  else disease_0 = 2//uncorrelated

Asterisk represents all suffix numbers of this type of attribute.

In the personal history, only the attributes of smoking, years of smoking (smoking_year), and smoking amount (smoking_value) are considered, and they are reduced to an attribute smoking_0. The attribute values 1, 2, and 3 represent high value and long time, high value and short time, and low value and long time, low value and short time, and no smoking, respectively. The logical relationship of the attribute smoking_0 was given as follows:

  if (smoking_year = 0 and smoking_value = 0) then smoking_0 = 5
  else if smoking_year >10 then
  if smoking_value > 1 then smoking_0 = 1
  else smoking_0 = 3
  else if smoking_value > 1
  then smoking_0 = 2
  else smoking_0 = 4

Some redundant attributes in the original data table can be deleted directly (for example, the attribute of drinking in personal history).

### 2.5. Collection of Research Data Related to Psychological Conditions of Patients

The research data related to the psychological conditions of patients were collected, and the main research tools used included the questionnaire on personal basic information, *General Self-Efficacy Scale* (GSES), and *Social Support Scale*. A total of 168 patients participated in this study. The questionnaire on personal basic information is independently researched and compiled by the researcher. It mainly collects the sociodemographic statistics and general health status of patients, including gender, age, occupation, education level, economic level, marital status, payment method, department, hospitalization frequency, disease history, length of hospitalization, and comorbidities. The *Social Support Scale* covered a total of 13 items in three dimensions: objective support, subjective support, and utilization of social support.

### 2.6. Data Association Analysis

The Apriori algorithm was applied for data association analysis. The basic principle of the Apriori algorithm is to iterate successively and continuously scan the transaction database to find all frequent item sets that meet the requirements. It only scans the item sets with the same length each time, which is named as *K*-items set (*K* gradually increases from 1). *K* + 1 items are searched through *K* item sets, that is, low-level item sets are the basis of high-level item sets. The specific process is described as follows. Firstly, the database is scanned to mark the number of occurrences of all candidates, which is recorded as the support. Then, the items that are greater than or equal to the set minimum support are selected to form a frequent 1-item set L1. After that, the frequent 1-item set self-continuity is performed as a candidate frequent 2-item set C2. Next, the database is scanned again to mark the support of all candidate 2 item sets in C2, and the item set greater than or equal to the preset minimum support is selected as the frequent 2-item set L2. Such process should be repeated until there are no frequent item sets. The pseudocode representation process is shown in Table 1.

The Apriori algorithm has to scan the database every time when it looks for frequent sets, which leads to inefficiency. To solve this problem, the following two properties were adopted to compress the search space. Property 1: the necessary condition for the K-dimensional data item set *X* to be a frequent item set is that all its *K*−1 dimensional subsets are frequent item sets; property 2: if any (*t*−1)-dimensional subset of K-dimensional frequent item set *X* is not frequent item sets, then *X* is not the frequent item set either. The analysis of influencing factors related to the psychological status of patients is the same as the above method.

### 2.7. Statistical Analysis

The SPSS21.00 was adopted to perform statistical analysis on the collected data, with the chi-square test for count data and mean ± standard deviation $\left(\bar{x}\pm s\right)$ for measurement data. If the data distribution conformed to the normal distribution, the *T* test method was adopted. If the data distribution did not conform to the normal distribution, the nonparametric test method was adopted. If any indicator was compared within the group before and after treatment and the normal distribution conformed to the normal distribution, the *T* test was applied, or otherwise the *R* test was adopted. Data comparison between groups before and after treatment was performed by nonparametric test. The difference was statistically significant with *P* < 0.05.

## 3. Results and Discussion

CKD is defined as damage to the structure and function of the kidney caused by various reasons and the damage lasts for more than 3 months [13]. The disease has the characteristics of high incidence, high mortality, low awareness, and poor prognosis. Therefore, it has seriously threatened the lives and health of people for a long time. In recent years, the incidence of the disease has been further increased with the continuous increase of lifestyle changes, the intensification of population aging, environmental pollution, and drug abuse [14]. Therefore, early diagnosis and treatment of CKD to delay its development into end-stage renal disease is very urgent and necessary. At present, the treatment of CKD is very limited by western medicine. Diet control is the foundation, and then active control of the primary disease can avoid the further development of factors that damage the kidneys and the emergence of complications [15]. In addition, dialysis treatment is performed in the middle and late stages of the disease. This is the basic idea of the current western medicine treatment of chronic nephritis. At present, researches related to western medicine are mostly focused on the prevention and treatment of various complications. There are few studies on conservative treatment in internal medicine [16]. In general, there is currently no particularly effective treatment. Clinically, the treatment of CKD still has many defects, such as many complications and poor patient compliance. It is necessary to further study so as to find an exact and effective treatment plan [17]. Using the data mining technology, this study summarized and explored the clinical diagnosis and treatment of CKD on the basis of electronic records. The results were as follows.

### 3.1. General Data of Patients

The electronic medical records of 168 patients were collected, with 876 visits. The basic data of patients are shown in Figures 1∼5, including the age, gender, primary disease, and complications.  Figure 1 illustrates that the minimum age of patients was 23 years, the maximum age was 88 years, and the average age was 65.1 ± 15.011 years. There were 6 people aged 20–30 years (5%), 7 people aged 31–40 years (5%), 16 people aged 41–50 years (12%), 22 people aged 51–60 years (17%), 32 patients aged 61–70 years (24%), 35 people aged 71∼80 tears (25%), and 14 people older than 80 (11%). As given in Figure 2, there were 86 cases with chronic renal insufficiency (70%), 10 cases with hypertension nephropathy, 14 cases with nephrotic syndrome, 6 cases with chronic nephritis, 4 cases with purpuric nephritis, and 3 cases with IgA nephropathy according to the diagnosis results of western medicine. Analysis on Figure 3 suggests that there were 66 people with hypertension disease, 44 people with diabetes, 35 people with hyperlipidemia, 22 people with hyperuricemia, 19 people with osteoporosis, and 12 people with CHD. As illustrated in Figure 4, the numbers of patients accompanied with renal anemia, renal bone disease, constipation, and insomnia were 15, 11, 10, and 6, respectively. Analysis of Figure 5 shows that, in the 886 visits, 585 of 674 weaknesses were improved (87.8%), 418 of 490 back pains were bettered (86.6%), and 359 of 362 visits due to edema were improved (96.5%).

### 3.2. Analysis of Patient Symptoms and Signs

The frequency analysis method was adopted to analyse the symptoms and signs of 127 CKD patients; the symptoms with incidence greater than 3% are summarized in Table 2. It showed that back pain was the symptom with the highest incidence (35.11%), and the incidences of edema, backache, and waist distension were relatively high.

### 3.3. Cause Analysis

The etiology distribution of the patients is shown in Figure 6. Analysis of Figure 6 shows that there were 128 patients, and the most common causes were chronic glomerulonephritis, aristolochic acid nephritis, diabetic nephritis, and hypertensive nephritis, with the frequency of 442 times, 165 times, 130 times, and 117 times, and the rates of 43.76%, 16.34%, 12.87%, and 11.58%, respectively.

### 3.4. Time for Patients with Different Etiologies Developing Renal Failure

Figure 7 shows the statistical results of the time from the diagnosis of the primary disease to the first diagnosis of renal failure in patients with different etiologies. It illustrated that the average time for patients with chronic glomerulonephritis to be diagnosed with renal failure was 10.09 ± 5.99 years, that for patients with diabetic nephropathy was 10.99 ± 4.44 years, and that for patients with hypertension nephropathy was 12.99 ± 9.98 years. In addition, patients with aristolochic acid nephropathy were in the renal failure stage at the time of diagnosis.

### 3.5. Incidence of Hypertension

Hypertension is defined as systolic blood pressure (SBP) ≥140 mmHg, diastolic blood pressure (DBP) ≥90 mmHg, or the case requiring taking antihypertensive drugs to control blood pressure. The statistical results of hypertension in patients at different stages and causes are shown in Figure 8. It revealed that the overall incidence of hypertension was 80.4%. The incidences of renal function compensatory hypertension, renal function decompensated hypertension, renal failure phase hypertension, and uremia phase hypertension were 81.8%, 75%, 78%, and 84.4%, respectively. Therefore, there was no statistical difference in the incidence of hypertension in different periods (*P* > 0.05).

As given in Figure 9, the incidence of hypertension in patients with chronic glomerulonephritis, diabetic nephropathy, aristolochic acid nephropathy, nephropathy, and hypertension was 80.2%, 86.4%, 79.9%, and 100%, respectively. Therefore, the incidence of hypertension for patients with different primary disease was not statistically obvious (*P* > 0.05).

### 3.6. Incidence of Anemia

The statistical results of the incidence of anemia in patients at different stages and causes are shown in Figures 10 and 11.  Figure 10 shows that the overall incidence of anemia was 91.1%. The incidence of anemia for patients with compensatory renal function, decompensated renal function, renal failure, and uremia was 91.1%, 51%, 81.3%, 97.7%, and 99.2, respectively. There were statistical differences in the incidence of anemia in different periods (*P* < 0.05).

As revealed in Figure 11, the overall incidence of anemia in patients with different primary disease types was 91.1%. The incidence of anemia in patients with aristolochic acid nephropathy, diabetic nephropathy, chronic glomerulonephritis, and hypertension nephropathy was 97.2%, 96.8%, 88.9%, and 79.3%, respectively. It suggested that the incidence of anemia for patients with the four primary disease patients was relatively high with slight differences.

### 3.7. B-Ultrasound Results of Kidney

B-ultrasound of kidney is the most commonly used examination method for CKD. The kidney size of patients with different etiologies at different times was analysed in this study, and the analysis results are shown in Table 3. Comparison on the kidney size of patients with four causes showed great differences in the left and right long axis (*P* < 0.05), the left and right short axis (*P* < 0.05), and the left and right cross-sectional area (*P* < 0.05). In each group of data, the values of diabetic nephropathy were the highest, and the values of *Aristolochia* nephropathy were the smallest. B-ultrasound comparison of the kidneys in the groups showed that the left and right short axis and the left and right cross-sectional areas of the chronic glomerulonephritis group were statistically different (*P* < 0.05), and the left kidney was larger than the right kidney. There were remarkable differences in the left and right long axis, left and right short axis, and left and right cross-sectional areas of *Aristolochia* nephropathy (*P* < 0.05), and that in the left kidney was larger than the right one.

For the treatment of hypertension in CKD patients, the commonly used treatment method is oral antihypertensive drugs. Among 168 patients, a total of 144 patients underwent antihypertensive treatment during hospitalization. Six drugs were adopted, including angiotensin-converting enzyme inhibitors (ACEI), angiotensin receptor blockers (ARB), *β*-block, Ca ion antagonists (CCB), diuretics, and *α*-block. The CCB was the most widely used. 80% of patients received combination therapy, and the detailed usage is shown in Figure 12.

Erythropoietin (EPO) is the most commonly used drug for the treatment of anemia in CKD patients. In this study, a total of 155 patients had complete blood routine data, of which 138 patients used EPO. The detailed EPO usage is shown in Figure 13. It suggested that patients with hemoglobin less than 30 g/L and patients with hemoglobin within 60∼89 g/L used EPO the most.

For patients with advanced CKD, substitution therapy is the main treatment method. In this study, there were a total of 100 patients with uremia, of which 46 (46%) patients underwent the substitution therapy, including 26 patients (56.5%) on hemodialysis, 14 patients (32.6%) on peritoneal dialysis, and 5 cases (10.8%) on kidney transplantation (as given in Figure 14).

### 3.8. Factors Affecting Mental Health of Patients

CKD shows the characteristics of poor prognosis, complications, long course of disease, and more expensive treatment [18]. These characteristics lead to greater mental stress for patients, which further increases the possibility of patients suffering from mental illness. Depression is a common psychological and physical abnormal response that CKD patients often experience [19–21]. Once such emotion appears, the person is indifferent to the people or things around him, the appetite decreases, and the compliance decreases during the treatment and does not follow the doctor [22, 23]. In severe cases, there may even be suicidal tendencies, which is very unfavourable for the prognosis of the treatment of the disease. Previous studies have shown that pain and discomfort and neuroendocrine changes caused by chronic diseases cause changes in the transmitters of the central nervous system, thereby inducing the depression. Basically all patients with chronic diseases are accompanied by varying degrees of mental dysfunction, and the most frequent occurrence is depression [24–26]. All in all, mental illnesses and CKD recovery interact with each other. Relevant research results show that the incidence of depression in patients with chronic diseases is highly correlated with the course of disease, economic income, personality, and social support but shows low correlation with education level and age [27].

The age, gender, occupation, marriage, education level, economic income, medical expenses payment method, number of hospitalizations, and length of hospitalization of patients were undertaken as the influencing factors of the *Psychological Screening Inventory* (PSI) [28] score for analysis of variance. The results showed that the economic self-evaluation, income, education level, and disease history can meet the conditions of analysis of variance. The analysis showed that all variables were not statistically great (*P* > 0.05). Specific details are shown in Table 4.

In the univariate analysis, there was no obvious correlation between the general information and psychological status of patients. The general information was grouped into four items: economic self-evaluation, income, education level, and disease history. The Kruskal-Wallis H test [29] was performed on their groups, and the test results showed that there was no visible difference in the disease history and education level, but statistical differences were obvious in economic self-evaluation and income. The detailed results were shown in Table 5.

The correlation of the scores of the three factors of social support and the total support score to the psychological response score was analysed, and the results are shown in Table 6. It indicated that there was a significant correlation between the psychological status of patients and the three dimensions of social support and total support.

The three dimensions of coping styles, face, avoidance, and yield, were used as dependent variables to perform the regression analysis with the “enter” method. The analysis results revealed that avoidance and yield entered the regression equation, and the face was eliminated. This meant that avoidance and yield are greatly related to the psychological status of patients, as shown in Table 7.

### 3.9. Statistics of Mental Disease Intervention Models

At present, domestic and foreign scholars have conducted a lot of research on the treatment and intervention of the mental health of chronic patients. In addition to drug-based treatment, various psychological therapies play an important role in the treatment process. For example, some scholars have proposed three steps for psychological intervention for patients with chronic hospitalized depression: the first step is to listen to the patient's complaints and analyse the causes of depression; the second step is to give explanations, guidance, clarifications, and other psychological interventions based on the analysed reasons; and the third step is to comprehensively evaluate the effects of psychological intervention, analyse unresolved psychological problems, and further improve psychological intervention measures [28]. At present, the more common treatment methods include enhancing social support, changing coping styles, comprehensive psychological intervention, and effective health guidance. However, the research on mental health in our country started relatively late, and the people's awareness and attention to mental health are not high. Related research is relatively lagging [29]. This article sorted out and summarized the common psychological treatments and their effects for patients with clinical chronic kidney disease in China. The details were as follows:

98 of 168 patients in this study received psychological nursing intervention. The specific main intervention methods and patient depression scores before and after intervention are shown in Table 8. Analysis of Table 8 shows that there was no significant difference between the depression scores of the four groups of patients before the intervention. After the intervention, the depression scores of the patients all decreased to different degrees, in particular, the depression scores of the patients after the target behavioural nursing and mindfulness therapy intervention were significantly lower than those before the intervention, and the difference was statistically significant (*P* < 0.05).

## 4. Conclusions

The data mining technology was adopted on the basis of electronic medical records in this study to explore the rules of clinical diagnosis and treatment of CKD and the influencing factors on mental health of patients. It was found that the common symptoms of CKD patients were back pain, thirst, weakness, poor sleep, and so on. The most common primary diseases of CKD were chronic glomerulonephritis, aristolochic acid nephritis, diabetic nephritis, and hypertensive nephritis. The four primary disease patients were more prone to anemia and hypertension, and the kidney size under B-ultrasound was different. There were mental illnesses in the patients to a certain extent, which suggested that, in the clinical care of CKD patients, there are more encouragement and guidance of patients to actively face the disease. This study could provide a reference and basis for the further development of the treatment of CKD and the exploration of clinically relevant mental illnesses nursing intervention models. Due to the limited sample and scope, there may be some errors in the research results of this study. In the future study and work, it will further expand the sample size and scope of the research for comprehensive and in-depth research.

## Figures and Tables

**Figure 1:** Age distribution of patients.

**Figure 2:** Counts of primary diseases of patients.

**Figure 3:** Counts of complications of patients.

**Figure 4:** Counts of accompanied symptoms.

**Figure 5:** Statistical results on major symptoms of patients. (a) Frequency; (b) improvement rate.

**Figure 6:** Pie chart of the etiology distribution of patients.

**Figure 7:** Time for patients with different etiologies developing renal failure.

**Figure 8:** The incidence of hypertension in patients at different disease stages.

**Figure 9:** The incidence of hypertension in patients with different primary diseases.

**Figure 10:** The incidence of anemia in patients at different stages. *Note*. ^*∗*^ meant the difference was statistically obvious in contrast to the incidence of anemia for patients with compensatory renal function.

**Figure 11:** The incidence of anemia in patients with different primary diseases.

**Figure 12:** Drug usage for treatment of hypertension in CKD patients. (a) Types of applied oral antihypertensive drugs; (b) percentage of patients with combination therapy.

**Figure 13:** The detailed EPO usage for patients.

**Figure 14:** Number of patients who received substitution therapy.

**Table 1:** Pseudocode representation of Apriori algorithm process.

Input:
I//item-sets
D//affair dataset
S//support
Output:
L//item-sets
Process of the Apriori algorithm:
*K* = 0://K means the times of scanning
*L* = Φ:
Ci = I://the initial candidate set is set to a single item
Repeat
*K* = K + 1:
Lk = Φ:
For each Ii⊂Ck do
Ci = 0://the initial data of each item set is set to 0
For each tj⊂D do
For each Ii⊂Ck do
If Ii⊂tj then
Ci = Ci + 1:
For each Ii ⊂Ck do
If Ci ≥ (S × D) then
Lk = Lk∪Ii:
*L* = L∪LK:
CK + 1 = Apriori-Gen (LK)
Until Ck + 1 = Φ

**Table 2:** Statistical results of patient symptoms and signs.

No.	Symptoms	Incidence (%)
1	Back pain	35.11
2	Thirst	35.03
3	Weakness	31.22
4	Poor sleep quality	25.9
5	Frequent urination at night	25.11
6	Edema	24.8
7	Backache	16.15
8	Dizzy	15.66
9	Waist pain	13.88
10	Fear of the cold	13.46
11	Itchy skin	13.19
12	Bitter	12.01
13	Reduced appetite	11.33
14	Dry stool	8.66
15	Dreaminess at night	8.49
16	Easy to catch a cold	8.49
17	Cough	7.58
18	Sputum	6.98
19	Nausea and retching	6.88
20	Thin stools	6.11
21	Increased frequency of urination	5.81
22	Abdominal pain	5.78
23	Joint pain	5.88
24	Numbness in limbs	5.67
25	Tired	4.91
26	Chest tightness and shortness of breath	4.91
27	Swollen limbs	4.28
28	Stomach pain	4.18
29	Stomach pain	3.79
30	Tight breathing	3.29
31	Diarrhea	3.11
32	Fatigue and weakness	3.09

**Table 3:** Comparison on kidney size of patients with different courses.

Item	Chronic glomerulonephritis	Diabetic nephropathy	Hypertensive nephropathy	*Aristolochia* nephropathy
Left and right long axis (cm)	8.83 ± 1.02^*∗#*^	9.53 ± 0.88^*∗*^	8.32 ± 1.18^*∗#*^	7.56 ± 0.77^*#&*^
Long axis of right kidney (cm)	8.72 ± 0.91^*∗#*^	9.35 ± 0.53^*∗*^	8.33 ± 1.05^*∗*^	7.23 ± 1.21^*#*^
Short axis of left kidney (cm)	4.42 ± 0.52^*∗&*^	4.36 ± 0.46^*∗*^	4.13 ± 0.71^*#*^	3.76 ± 0.35^*#&*^
Short axis of right kidney (cm)	4.33 ± 0.76^*&∗#*^	4.62 ± 0.35^*∗*^	4.18 ± 0.65^*∗*^	3.53 ± 0.44^*#*^
Left renal cortex (cm)	1.17 ± 0.42	1.2 ± 0.3	1.2 ± 0.3^*∗*^	1.1 ± 0.4
Right renal cortex (cm)	1.08 ± 0.55	1.3 ± 0.2^*∗*^	1.3 ± 0.5	1.1 ± 0.4^*#*^
Left kidney area (cm^2^)	37.27 ± 8.66^*∗#&*^	43.96 ± 7.79^*∗*^	35.16 ± 8.36^*∗#*^	30.55 ± 6.38^*#&*^
Right kidney area (cm^2^)	34.53 ± 9.39^*∗#*^	44.02 ± 6.38^*∗*^	35.82 ± 9.07^*∗*^	28.37 ± 5.43^*#*^

*Note*. ^*∗*^, ^*#*^, and & indicate that the difference satisfied *P* < 0.05 in contrast to the *Aristolochia* nephropathy, diabetic nephropathy, and right kidney, respectively.

**Table 4:** Correlation between general information and psychological status of patients.

Variable	F	*P*
Gender	2.477	0.117
Age	0.24	0.877
Occupation	0.744	0.66
Marriage	0.588	0.711
Payment	2.112	0.099
Number of hospitalizations	0.850	0.355
Length of hospitalization (days)	1.466	1.466
Combined diagnosis	0.763	0.384

**Table 5:** Nonparametric test results of rank conversion.

Variable	H	*P*
Economic self-evaluation*∗*	21.775	*P* ≤ 0.001
Income*∗*	26.122	*P* < 0.001
Education level	4.211	0.123
Disease history	4.113	0.259

*Note.* ∗ means *P* < 0.001, showing statistical significance.

**Table 6:** Correlation between social support and psychological status of patients.

*r*	Subjective	Objective	Utilization	Total support
Psychological status	−0.127^*∗*^	−0.074^*∗*^	−0.109^*∗*^	−0.142^*∗*^

*Note.* ^*∗*^ means *P* < 0.05.

**Table 7:** Correlation between attitudes towards diseases of patients and their mental states.

Dependent variable	Independent variables	B	Beta	*t*	*P*
Psychological status	Face	0.274	0.038	1.086	0.277
	Avoidance^*∗*^	0.789	0.096	2.792	0.005
	Yield^*∗*^	4.276	0.380	10.866	*P* ≤ 0.001

*Note*. ^*∗*^ means *P* ≤ 0.001, showing statistical significance.

**Table 8:** Depression scores of patients before and after different psychological interventions.

Intervention method	Cases	Before intervention	After intervention	*P*
Psychological counseling therapy	33	50.48 ± 9.32	49.21 ± 10.01	0.18
Target behaviour care	27	52.21 ± 8.12	48.01 ± 9.33	0.032
Music therapy	21	51.13 ± 8.84	49.09 ± 9.11	0.051
Mindfulness intervention	17	50.99 ± 9.77	47.01 ± 9.33	0.024

## Data Availability

The data used to support the findings of this study are available from the corresponding author upon request.
